# Mental Health Study from the Perspective of Behavior Preference under the Environment of Internet Media: Based on China's Data Analysis

**DOI:** 10.1155/2022/2523093

**Published:** 2022-09-27

**Authors:** Guangjun Chen, Yubo Zhong, Wangyang Yu, Jin Yan

**Affiliations:** ^1^Xingcheng Teaching Base, Jilin University, Huludao, Liaoning 125000, China; ^2^Jilin University College of New Energy and Environment, Changchun, Jilin 130012, China; ^3^Office of the CPC Committee, Beijing Normal University, Beijing 100875, China; ^4^Foreign Languages College Changchun University, Changchun, Jilin 130022, China

## Abstract

To prevent the mental health problems of college preference students effectively, this paper analyzes the influence of college students' internet media use behaviors on their mental health in the information age. We make an empirical study on the above problems by using metrology models under the condition of controlling individual factors. The result shows that the mental health of college students is significantly affected by different internet media use behaviors and shows obvious heterogeneity. Preference for games and soap operas or films has a significant negative relationship with the mental health of college students, while the preference for science, education programs, and the preference to obtain current political news comments through official media have a positive impact on the psychological security of college students. Meanwhile, the mental health of college students is also significantly influenced by individual factors. The education level, family income, and social satisfaction show a significant positive correlation with the mental health of college students.

## 1. Introduction

Safety needs are a basic human need. For college students, physical safety guarantees their external physical health, but if their mental health needs are not met, it will endanger their physical and mental health and affect their overall development. If a person has mental health problems, there is no real health [1]. Therefore, the importance of mental health education in colleges and universities is self-evident. Generally speaking, the content of mental health education for college students should include all aspects of college life such as outlook on life and values, formation of self-awareness, personality development, study habits and abilities, interpersonal interactions, love and sexual psychology, emotional experience and control, requirements for facing frustration, job hunting, psychological testing and assessment, and psychological counseling and psychotherapy [2, 3]. In China, mental health education in colleges and universities has made great progress in recent years, with more comprehensive mental health standards, gradually improved mental health education curriculum construction, more mental health lectures and mental health counseling [4], and a growing faculty. According to a recent study by Kim and Hong [5], Chinese college students' mental health education covers many aspects of health concepts, self-awareness, interpersonal interaction, learning, personality, emotion, frustration, psychosexuality, love, internet, career choice, counseling, and psychotherapy. At the present stage, mental health education in Chinese universities has shown a good development trend. However, it is undeniable that there are still many shortcomings in the mental health education of Chinese college students, which faces a series of problems, such as low attention, lagging construction of software and hardware supporting facilities, large regional differences in mental health education, and the lack of specialization, professionalism, and expertism of university student mental health education teachers, which seriously hinder the effective intervention of university students' psychological problems.

Mental health problems among college students have become a global public health issue. Most psychological problems first appear in early adulthood, especially between the ages of 17 and 24 [6, 7]. Some studies have shown that the prevalence of mental disorders among youth groups ranges from 8.3% to 12.4% [8], and evidence can be found in the undergraduate group [9]. In recent years, the psychological problems of college students around the world have been increasing. A large percentage of college students meet the criteria for different psychological disorders during their college years [10]. In the United States, according to the Healthy Minds Study, the prevalence of depression among college students was found to be 39% and 34% for anxiety disorders [11]. In Chile, South America, the prevalence of mental health problems among college students has increased over the past few years [12]. The prevalence of depression and anxiety among Chilean college students was as high as 46% in 2019 [13].

According to relevant studies, the mental health problems among Chinese college students have become increasingly complex and are on the rise [14, 15]. At present, about 30% of college students in China suffer from different degrees of mental illness, and 33.3% of them have more serious mental illnesses [16]. In recent years, the phenomenon of college students dropping out of school and suicide due to mental illness has become more and more common [17]. In order to analyze the demand for mental health services of Chinese college students, a researcher analyzed the demand for mental health services in 35 colleges and universities and 5058 college students in China by means of a questionnaire. And the study found that contemporary Chinese college students have a high demand for mental health services [18]. Most college students are eager to receive mental health services from school mental health education centers, community psychological support centers, and company psychological service centers. Specifically, female college students have significantly higher needs for mental health services than male college students, and freshman and senior year college students have significantly higher needs for mental health services than sophomore and junior year college students [19]. The mental health status of college students and the initiatives taken by colleges and universities to respond to college students' mental health problems have become the focus of social attention [20].

Existing research mainly adopts questionnaires, interviews, and theoretical analysis to explore the causes of mental health problems affecting college students from the perspectives of online media interaction, preference of media use and online games. There are few relevant research topics and a single research method, which makes the research conclusions lack persuasive power. This study explores the factors influencing the mental health problems of college students in the new media era more accurately through empirical analysis using the Chinese Internet users' social awareness survey database. And the marginal contributions of this paper are mainly in the following aspects. First, compared with analysis methods such as questionnaires and interviews with small samples, this paper uses data at the database level to conduct analysis and draw more convincing conclusions in the context of big data. Second, this paper explores the causes of college students' psychological problems from multiple perspectives, which makes the factor analysis more comprehensive. In addition, the rest of the paper is organized as follows. The second part is the part of theoretical analysis and research hypothesis. The third part is the analysis of college students' mental health index measurement and evaluation. The fourth part is the part of empirical analysis. And the fifth part is the conclusion and policy suggestion part.

## 2. Theoretical Analysis and Research Hypothesis

Mental health of an individual usually shows that the individual has no fear, does not worry about the accusation and criticism of others, and maintains a safe, free, solid, and stable psychological state inside. The ideal psychological health of college students is usually characterized by optimistic and positive emotions, normal intellectual level, harmonious interpersonal relationships, stable and appropriate emotions, mature and appropriate behavior, correct cognition, good personality quality, and strong will. The mental health problems of college students mainly originate from a series of physical and mental pressures they face, which mainly come from social responsibilities, life itself, competitive pressures, the fast pace of social progress, etc. The external reason is often that their mental health problems do not attract enough attention and do not receive timely and professional psychological intervention. The mental health problems of contemporary college students are mainly manifested as anxiety, autism, depression, paranoia, compulsion, irritability, schizophrenia, thought disorders, and other problems caused by weak environmental adaptability, incompatible interpersonal relationships, unsatisfactory grades, and complex emotional problems. Today, depression, anxiety, eating disorders, and other symptoms of mental illness are becoming more prevalent in the college student population and are a mental health crisis that society as a whole society has to pay attention to. Therefore, it is imperative to conduct scientific research and seek possible solutions to meet the mental health needs of college students [21].

Specifically, the factors influencing the mental health of college students can be broadly classified as self, family, school, and social factors [22–26]. Among them, the main factors of self are gender, the origin of the student, major medical history, major, satisfaction with an application, student cadre experience, academic performance, and self-care ability. Family factors mainly include early childhood upbringing, family structure, family atmosphere, family economic status, and other factors [27, 28]. School factors mainly include learning environment, dormitory environment, curriculum arrangement, teacher-student relationship, ideological and political education, and the importance of mental health teaching. The main social factors are social atmosphere, social competition pressure, and the impact of diversified network information. From the existing empirical studies, it can be found that there are differences in interests, emotions, interpersonal relationships, social adaptation, competitiveness, and innovative thinking among college students, influenced by factors such as gender, grade, academic performance, and major, which in turn have an impact on the mental health of college students. Specifically, the level of psychological quality of freshman and sophomores changed less, the psychological quality of juniors showed a decreasing trend, the psychological quality of seniors fluctuated more, and academic performance was positively correlated with the psychological quality of college students [29, 30]. And the psychological quality of college students varied among majors. In addition, the study tasks, professional interests, average daily Internet time, and Internet age of college students also have a strong correlation with mental health problems of college students. The study found that the mental health of college students from urban areas with harmonious family relationships was significantly higher than that of college students from rural areas with poor family relationships, and the mental health of students who were satisfied with their majors had no study pressure or less pressure and had less employment pressure was relatively better. Based on the above analysis and also combined with the characteristics of Chinese Internet users' social awareness survey data, the hypotheses can be proposed.

**Hypothesis 1 .**

Individual characteristics such as education level, family income level, and social satisfaction can have a positive impact on the mental health of college students.

It is worth noting that the emergence of new online media with the Internet and smartphones as the platform makes people's communication more convenient, which has greatly satisfied the diverse needs of college students' cognitive development. Among them, science and education programs mainly focus on human history, scientific exploration, and cultural education. Taking the CCTV Science and Education Channel as an example, it always takes “educational character, scientific quality, and cultural taste” as its core concept and refuses to vulgarize entertainment programs, fully satisfying the audience's need to acquire knowledge, opinions, and ideas. The official authoritative website shoulders the social mission of promoting positive energy, and the report content has strong rigor, authority, and credibility. Science and education educational resources and official authoritative reports can not only lay a good professional and technical foundation for the future development of college students but also help them develop a correct worldview, outlook on life and values, guide them to establish positive ideas and beliefs, and help them establish a positive outlook for the future, and good expectations for the future can have a positive impact on college students' mental health and even “happiness for the rest of their lives” [31]. Scientific and cultural knowledge and correct emotional values conveyed by official authoritative reports are largely conducive to cultivating self-confidence, forming good expectations, becoming more optimistic, and strengthening mental toughness [32]. That is conducive to the accumulation of psychological capital of college students. According to relevant studies, psychological capital has been found to be effective in relieving people's work stress and fatigue [33] and can also actively help people to improve life satisfaction, happiness, sense of belonging, and better behavioral performance [34–36]. Therefore, based on the above analysis, we propose the following hypothesis.

**Hypothesis 2 .**

College students' online media use behavior preference has a significant impact on college student's mental health and has heterogeneity characteristics.

**Hypothesis 3 .**

The preference of science and education programs and the preference of using authoritative official media channels to obtain news behavior have a positive effect on the mental health status of college students.

Of course, the new media era also provides a complicated virtual world for college students, such as various soap operas and online games, which are full of various bad culture and garbage information, which not only adversely affect the normal study and life of college students but also may make college students addicted to the virtual world for a long time and bring greater stimulation to physical strength, eyesight, and psychological aspects. According to the stimulus-organism response theory, changes in an individual's internal emotional state upon stimulation trigger a series of responses [37]. According to this theory, most information about changes in the environment is transmitted to the individual's nervous system, which in turn stimulates a series of muscular or psychological responses [38]. Therefore, the abovementioned series of bad stimuli are highly likely to make college students form unhealthy lifestyles and develop negative attitudes toward life and also have extremely negative effects on their self-efficacy and social responsibility. Lifestyle [39], attitude toward life [40], self-efficacy [21, 41], and social responsibility are closely related to the mental health of college students.

In addition, undesirable information and cybercrime in the Internet seriously threaten the physical and mental safety of college student groups and are very likely to lead to cognitive confusion, personality disorders, weakened self-discipline, social disorders, and Internet addiction, which in turn lead to a series of mental health problems such as irritability, anxiety, and personality distortion, have an extremely negative impact on interpersonal interactions and normal behavioral norms of college students, and can easily trigger college students' psychological violence [42–44]. Psychological violence-induced depression [45], traumatic stress disorder [46], decline in academic performance [43, 47, 48], and trauma have a negative impact on both their own and others' mental health. Therefore, the following research hypotheses can be put forward.

**Hypothesis 4 .**

Soap operas, romantic drama-type behavioral preferences, and online game behavioral preferences have a negative impact on college students' mental health status.

## 3. Measurement and Statistical Analysis

### 3.1. Data Source and the Description of Indicators

The mental health of college students generally refers to a good or normal coping psychological mechanism in the face of the internal and external environment, which usually manifests itself in positive and stable emotions, harmonious interpersonal relationships, scientific and standardized cognition, good personality, and strong will. This paper combines the basic characteristics of college students' mental health, and also in view of the availability of data, this paper selects the indicators of being critical and argumentative (Q1), being poorly organized and careless (Q2), being emotionally stable and calm in situations (Q3), having a plan and being efficient (Q4), having difficulty deciding what is really wanted in shopping (Q5), being usually quick and confident in making important decisions (Q6), being indecisive (Q7), and being indecisive in most decisions (Q8) from the 2017 Chinese Internet users' social consciousness survey database for a comprehensive reflection of college students' mental health. It should be noted that in the original database, indicators such as emotional stability, calmness (Q3), planning and efficiency (Q4), and making important decisions quickly and confidently (Q6) are high-optimality indicators, i.e., higher indicator scores indicate better mental health, while indicators such as criticism and quarreling (Q1), poor organization and carelessness (Q2), difficulty in deciding what is really wanted in shopping (Q5), indecisiveness (Q7), and indecisiveness in most decisions (Q8) are low-optimality indicators, i.e., lower indicator scores indicate better mental health. To make the indicators comparable, this paper further uses the linear interpolation method to transform the above low-quality indicators into high-quality indicators. In general, the above indicators can generally reflect the mental health status of college students in the 2017 Chinese Netizen Social Awareness Survey Database.

Since the research subjects of this paper are college students groups, including undergraduate and graduate students, the actual empirical data used need to be screened from the Chinese Netizen Social Awareness Survey Database. The specific screening process is as follows: first, the samples with the age group below 18 and above 35 are deleted. Second, only the samples with the occupation of “studying in school” are retained. After the data screening process, 458 valid samples were obtained, which is the basic sample data for the empirical analysis of this paper.  Table 1 gives a brief statistical description of the sample data in this paper. According to the statistical results in Table 1, there were 458 valid samples of sample data finally screened in this paper, among which 157 were male, accounting for 34.28% and 301 were female, accounting for 65.72%; 314 were undergraduates, accounting for 68.56% and 137 were masters, accounting for 29.91%.

In the empirical study of the influence of college students' media use behavior on mental health, there is no single fixed indicator to measure mental health because it involves multiple dimensions. Therefore, in order to reflect the mental health problems of college students in a comprehensive manner, several mental health-related indicators must be considered in an integrated manner. In the Chinese Netizen Social Awareness Survey Database (2017), the abovementioned Q1 to Q8 question items all reflect certain information of college students' mental health to different degrees. Therefore, it is better to include the information reflected by the above indicators when conducting the measurement of the mental health index of college students. In addition, too many variables in the empirical analysis of multivariate problems by statistical methods will not only increase the calculation volume but also increase the difficulty and complexity of the analyzed problems. We found that there were strong correlations among the above eight question items reflecting college students' mental health, and the information overlapped to some extent. Therefore, the idea of dimensionality reduction can be used to reduce multiple variables into fewer variables. And the factor analysis method is a commonly used ideal tool for dimensionality reduction of indicators.

### 3.2. Mental Health Index Measurement of College Students

We analyzed the correlations of the question items from Q1 to Q8 to make a preliminary judgment on whether it is reasonable to use the factor analysis method.  Table 2 gives the correlation coefficient matrix of the indicators related to college students' mental health.

The applicability of the factor analysis method in this paper was further judged by KMO and Bartlett test. In general, when the KMO value is greater than 0.70, it can be considered suitable for factor analysis. In addition, if the significance level corresponding to the chi-square statistic of Bartlett's spherical test is less than 0.01, it means that factor analysis can be done. If the null hypothesis is not rejected, it means that these variables may provide some information independently and are not suitable for factor analysis.  Table 3 presents the KMO and Bartlett test results. According to Table 3, the value corresponding to the KMO test is 0.77, which is greater than 0.70, and the significance level corresponding to the chi-square statistic of the Bartlett test is 0.00, which is less than 0.01. The test results show that it is more appropriate to use the factor analysis method to calculate the mental health index of college students based on the above indicators. The following is a factor analysis of the above seven indicators that comprehensively reflect the mental health of college students, and the principal component method is used to extract common factors. According to the eigenvalues and variance contribution rates of principal components in Table 4, three principal components with eigenvalues greater than 1 were extracted; the corresponding three eigenvalues were 2.988, 1.241, and 1.016; and the cumulative variance contribution rate reached 65.56%, that is, the three principal components retain most of the information of nearly 70% of the original indicators. In general, the three extracted principal components can be used to replace the original variable set.

### 3.3. Statistical Analysis of the Distribution of College Students' Mental Health Index

Based on the three principal component scores calculated by SPSS.22 software, multiply each principal component score by the corresponding weight *W* to get the comprehensive score of college students' mental health index. The principal component score weight *W* is the proportion of the eigenvalues corresponding to each principal component to the sum of the three eigenvalues.  Figure 1 below shows the distribution of Chinese college students' mental health index scores. As shown in Figure 1, the average value of the mental health index of Chinese college students is 0.00, the minimum value is 1.81, and the maximum value is 1.61. In addition, from the frequency distribution of college students' mental health index, there are relatively many college students whose mental health index is lower than the average. Specifically, in the 458 samples, 51.53% of the individual mental health index levels were lower than the average, while 48.47% of the individual mental health index levels were higher than the average.

## 4. Research Design and Analysis

### 4.1. Regression Model and Variable Descriptions

To empirically test the impact of college students' online media use behavior preference on mental health, this part conducts an empirical test by constructing multiple linear regression equation models. Combined with the previous analysis and practical experience, the following multiple linear regression model is constructed:

(1) $$\begin{array}{c} I=cons+\underset{i}{\sum }\gamma_{i}z_{i}+\underset{i}{\sum }\beta_{i}x_{i}+\varepsilon . \end{array}$$

#### 4.1.1. Dependent Variable

The explained variable in this paper is represented by *I* which is the mental health index of college students, and the mental health index of college students is calculated by the factor analysis method in the previous article. The higher the mental health index is, the better the mental health level is. And the smaller the mental health index is, the lower the mental health level.

#### 4.1.2. Independent Variable

To comprehensively reflect the preference of college students' online media uses behavior, specific relevant indicators were selected as explanatory variables from the 2017 Chinese Netizen Social Awareness Survey Database that is indicators such as college students' various online media use behaviors were selected, which were denoted by *x*_*i*_. Among them, the *x*_1_ represents the preference for obtaining information from commercial portals such as http://Sina.com and http://Tencent.com. The *x*_2_ represents the frequency of online shopping. The *x*_3_ represents the frequency of watching entertainment, sports news, movies, and TV dramas. The *x*_4_ represents the preference for humanities and arts articles. The *x*_5_ represents soap operas, romantic dramas, or movie preference. The *x*_6_ represents the preference of science and education programs. The *x*_7_ represents the preference for buying newspapers to read current affairs news. The *x*_8_ represents the preference for current affairs news through the analysis reports of the current affairs of CCTV, Xinhua News Agency, and People's Daily. The *x*_9_ represents the preference for obtaining current affairs news through government affairs portal websites, Weibo, and WeChat official accounts. The *x*_10_ represents chatting with friends. The *x*_11_ represents playing games. The *x*_12_ represents viewing and downloading study and work materials. The *x*_13_ represents organizing blogs, photo albums, and handling emails. And the *x*_14_ represents watching WeChat Moments and WeChat group messages or chat.

#### 4.1.3. Control Variables

To improve the parameter estimation accuracy of the multiple linear regression model, other factors affecting the mental health of college students are selected as control variables, among which the control variables are individual attribute variables: as gender, education level, living area, family annual income, social satisfaction, etc., which were denoted by *z*_*i*_. Among them, the *z*_1_ represents gender, the 1 represents male, and the 2 represents female. The *z*_2_ represents education level. The *z*_3_ represents living area. The *z*_4_ represents annual household income. The *z*_5_ represents social satisfaction.

### 4.2. Multiple Linear Regression Model Estimation

To empirically analyze the influencing factors of college students' mental health in the new media era and to consider the robustness of the empirical analysis results, this paper uses the least squares method to perform stepwise regression estimation of the multiple linear regression model and further uses the great likelihood estimation method and the binary logistic stepwise regression method for robustness testing. In the binary logistic regression model, if the mental health index of individual college students is greater than the mean value, it will be assigned a value of 1, indicating that the corresponding sample individuals do not have mental health problems. If the mental health index of individual college students is less than the mean value, it will be assigned a value of 0, indicating that the corresponding sample individual has mental health problems. Stata15.0 statistical analysis software was used for estimation, and the empirical estimation results are shown in Table 5. Among them, model 1 is the estimation result of least squares regression, model 2 is the estimation result of least squares regression using robust standard error, model 3 is the estimation result of maximum likelihood, and model 4 is the estimated value of regression coefficient of the binary logistic model. Since model 1, model 2, and model 4 use the stepwise regression method, Table 5 only lists the estimated results corresponding to the variables that have a significant impact on the mental health of college students.

### 4.3. Regression Analysis

According to the estimation results in Table 5, it can be concluded that, in terms of individual factors, the level of education has a positive and significant effect on the mental health level of college students; according to the estimation results of model 3 and model 4, the level of family income has a positive and significant effect on the mental health level of college students; according to the estimation results of model 1, model 2, and model 3, the higher the satisfaction of college students with society, the higher the level of mental health. Except for the above indicators, other variables do not have significant effects on the mental health of college students. In summary, Hypothesis 1 is verified. According to the estimation results in Table 5, it can be considered that soap operas, romantic dramas (movies) preferences, and gaming behavior preferences are not conducive to the improvement of college students' mental health, and they can harm the mental health level of college students, while science and education program preferences and behavioral preferences for obtaining news through authoritative official media such as CCTV, Xinhua News Agency, and People's Daily can have a positive and significant impact on college students' mental health. In addition, from the estimated results of the control variables, the educational level has a positive and significant impact on the mental health level of college students. In summary, Hypotheses 2-4 are verified.

## 5. Conclusions and Policy Implications

This paper analyzes the impact of mental health of college students in the new media era at the theoretical and empirical levels. Based on the empirical analysis, we get the following conclusions.

First, the preference for network media use behavior can have a significant impact on the mental health of college students, and it shows obvious heterogeneity. At the same time, the mental health of college students is significantly affected by individual factors. Second, in terms of network media use behavior preference: foam soap opera preference and game preference have adverse effects on the mental health of college students. The preference for science and education programs and the preference for obtaining information through authoritative official media channels such as CCTV, Xinhua News Agency, and People's Daily can have a positive and significant impact on the mental health of college students. Third, in terms of individual factors, education level, family income status, and social satisfaction can have a positive and significant impact on the mental health of college students.

Based on the research conclusions, this paper has the following policy implications.

First, in the era of new media, colleges and universities should actively open new media network quality education courses, guide college students to avoid indulging in online games and bubble soap operas, positively guide college students to effectively use various new media network resources, appropriately encourage college students to develop the habit of watching scientific and educational programs, and promote the all-round development of college students' moral, intellectual, physical, and aesthetic.

Second, we should give full play to the advantages of family education. Among the family factors, parenting style has the greatest influence on individuals and affects college students' individual cognition and individual characteristics. Parents should pay attention to the quality of material and spiritual life of college students and avoid college students' overreliance on new media networks for emotional and affective venting.

Third, the network authorities should actively establish a safe and effective new media network mechanism, strengthen the construction of new media norms and legal system, purify the new media network space, promote the construction of a universal safety culture network platform and safety culture service platform, and provide a clean and comfortable new media network environment for the physical and mental healthy growth of college students. In conclusion, schools, society, families, and individuals should establish a stable linkage mechanism [49] and make concerted efforts to jointly improve the mental health of college students.

## Figures and Tables

**Figure 1:** Distribution of Chinese college students' mental safety index.

**Table 1:** Statistical description of the sample.

Variate	Undergraduate	Masters and doctorates	Other samples	Total
Male	102	50	5	157
Female	212	80	2	301
Total	314	137	7	458

**Table 2:** Correlation matrix of college students' mental safety indicators.

Index	*Q*_1_	*Q*_2_	*Q*_3_	*Q*_4_	*Q*_5_	*Q*_6_	*Q*_7_	*Q*_8_
*Q*_1_	1	0.137^∗∗∗^	0.144^∗∗∗^	-0.033	-0.029	0.018	0.052	0.104^∗∗^
*Q*_2_	0.137^∗∗∗^	1	0.320^∗∗∗^	0.321^∗∗∗^	0.157^∗∗∗^	0.226^∗∗∗^	0.191^∗∗∗^	0.266^∗∗∗^
*Q*_3_	0.144^∗∗∗^	0.320^∗∗∗^	1	0.356^∗∗∗^	0.112^∗∗∗^	0.273^∗∗∗^	0.247^∗∗∗^	0.252^∗∗∗^
*Q*_4_	-0.033	0.321^∗∗∗^	0.356^∗∗∗^	1	0.121^∗∗∗^	0.311^∗∗∗^	0.301^∗∗∗^	0.286^∗∗∗^
*Q*_5_	-0.029	0.157^∗∗∗^	0.112^∗∗∗^	0.121^∗∗∗^	1	0.279^∗∗∗^	0.398^∗∗∗^	0.471^∗∗∗^
*Q*_6_	0.018	0.226^∗∗∗^	0.273^∗∗∗^	0.311^∗∗∗^	0.279^∗∗∗^	1	0.501^∗∗∗^	0.518^∗∗∗^
*Q*_7_	0.052	0.191^∗∗∗^	0.247^∗∗∗^	0.301^∗∗∗^	0.398^∗∗∗^	0.501^∗∗∗^	1	0.734^∗∗∗^
*Q*_8_	0.104^∗∗^	0.266^∗∗∗^	0.252^∗∗∗^	0.286^∗∗∗^	0.471^∗∗∗^	0.518^∗∗∗^	0.734^∗∗∗^	1

Note: ∗∗∗ means the significance level is 1%, ∗∗ means the significance level is 5%, and ∗ means the significance level is 10%.

**Table 3:** KMO and Bartlett test.

KMO		0.77
Bartlett's sphericity test	Chi-square statistic	891.32
	Degrees of freedom	28
	Salience	0.00

**Table 4:** Principal components eigenvalues and variance contribution rate.

Constituent	Initial eigenvalue variance			Extract the load sum of squares			Rotational load sum of squares		
	Variance contribution rate %	Cumulative contribution rate %	Eigenvalues	Variance contribution rate %	Cumulative contribution rate %	Eigenvalues	Variance contribution rate %	Cumulative contribution rate %	Eigenvalues
1	2.988	37.355	37.355	2.988	37.355	37.355	2.414	30.17	30.17
2	1.241	15.507	52.862	1.241	15.507	52.862	1.774	22.18	52.35
3	1.016	12.698	65.560	1.016	12.698	65.560	1.057	13.21	65.56
4	0.760	9.495	75.055						
5	0.647	8.089	83.144						
6	0.587	7.334	90.479						
7	0.508	6.345	96.824						
8	0.254	3.176	100						

**Table 5:** Empirical regression estimation results.

Variable	Model 1	Model 2	Model 3	Model 4
Behavioral variables				
*x*_5_	-0.097^∗∗∗^	-0.097^∗∗∗^	-0.087^∗∗∗^	-0.343^∗∗∗^
	(-3.89)	(-3.81)	(-3.05)	(-3.89)
*x*_6_	0.094^∗∗∗^	0.094^∗∗^	0.087^∗∗^	0.331^∗∗∗^
	(2.72)	(2.50)	(2.08)	(2.71)
*x*_8_	0.073^∗∗^	0.073^∗∗^	0.071^∗^	0.361^∗∗∗^
	(2.16)	(2.10)	(1.82)	(3.01)
*x*_11_	-0.051^∗^	-0.051	-0.042	-0.190^∗^
	(-1.68)	(-1.67)	(-1.34)	(-1.78)
Individual variables				
*z*_2_	0.137^∗∗^	0.137^∗∗^	0.113^∗^	0.487^∗∗^
	(2.20)	(2.29)	(1.75)	(2.24)
*z*_4_	0.027	0.027	0.030^∗^	0.164^∗∗∗^
	(1.53)	(1.55)	(1.65)	(2.63)
*z*_5_	0.073∗∗	0.072^∗∗^	0.082^∗∗^	0.169
	(2.13)	(2.17)	(2.38)	(1.44)
Constant terms	-0.767^∗∗∗^	-0.767^∗∗∗^	-0.643^∗^	-2.174^∗∗^
	(-2.84)	(-2.84)	(-1.80)	(-2.17)
*Ll*	-418.54	-418.54	-416.46	-284.93
chi2			66.42	56.43
*r*2_*p*				0.09
*r*2	0.10	0.10		
*N*	452	452	452	452

Notes: the values in brackets are standard deviations. ∗∗∗, ∗∗, and ∗ indicate that the estimated coefficients are significant at the confidence levels of 1%, 5%, and 10%, respectively.

## Data Availability

The dataset can be accessed upon request.

## References

[1] WHO (2013). *Who depression is a common illness and people suffering from depression need support and treatment*.

[2] Marques S. S., Braidwood R. (2021). Impact of the coronavirus lockdown on older adolescents engaged in a school-based stress management program: changes in mental health, sleep, social support, and routines. *Children & Schools*.

[3] Niederkrotenthaler T., Laido Z., Kirchner S. (2022). Mental health over nine months during the SARS-CoV2 pandemic: representative cross-sectional survey in twelve waves between April and December 2020 in Austria. *Journal of Affective Disorders*.

[4] Cage E., Jones E., Ryan G., Gareth H., Leigh S. (2021). Student mental health and transitions into, through and out of university: student and staff perspectives. *Journal of Further and Higher Education*.

[5] Kim T. W., Hong H. J. (2021). Understanding university students’ experiences, perceptions, and attitudes toward peers displaying mental health-related problems on social networking sites: online survey and interview study. *JMIR Ment Health*.

[6] De Girolamo G., McGorry P. D., Sartorius N. (2019). *Age of Onset of Mental Disorders: Etiopathogenetic and Treatment Implications*.

[7] Kessler R. C., Angermeyer M., Anthony J. C. (2007). Lifetime prevalence and age-of-onset distributions of mental disorders in the World Health Organization’s world mental health survey initiative. *World Psychiatry*.

[8] Gustavson K., Knudsen A. K., Nesvag R., Knudsen G. P., Vollset S. E., Reichborn-Kjennerud T. (2018). Prevalence and stability of mental disorders among young adults: findings from a longitudinal study. *BMC Psychiatry*.

[9] Valdés J. M., Díaz F. J., Christiansen P. M. (2022). Mental health and related factors among undergraduate students during SARS-CoV-2 pandemic: a cross-sectional study. *Frontiers in Psychiatry*.

[10] Sharp J., Theiler S. (2018). A review of psychological distress among university students: pervasiveness, implications and potential points of intervention. *International Journal for the Advancement of Counselling*.

[11] Eisenberg D., Lipson S. K. (2020). *The healthy minds study - fall 2020 data report*.

[12] Álamo C., Antúnez Z., Baader T., Kendall J., Barrientos M., Ddl B. (2020). The sustained increase of mental health symptoms in Chilean university students over three years. *Revista Latinoamericana de Psicología.*.

[13] Barrera-Herrera A., San M. Y. (2021). Prevalencia de sintomatología de salud mental y hábitos de salud en una muestra de universitarios chilenos. *Psykhe*.

[14] Benton S. A., Robertson J. M., Tseng W. C., Newton F. B., Benton S. L. (2003). Changes in counseling center client problems across 13 years. *Professional Psychology: Research and Practice*.

[15] Pledge D. S., Lapan R. T., Heppner P. P., Kivlighan D., Roehilke H. (1998). Stability and severity of presenting problems at a university counseling center: a 6-year analysis. *Professional Psychology: Research and Practice*.

[16] Ochnik D., Rogowska A. M., Kuśnierz C. (2021). Mental health prevalence and predictors among university students in nine countries during the COVID-19 pandemic: a cross-national study. *Scientific Reports*.

[17] Nottage M. K., Oei N. Y., Wolters N. (2022). Loneliness mediates the association between insecure attachment and mental health among university students. *Personality and Individual Differences*.

[18] Moore B., Dudley D., Woodcock S. (2019). The effects of martial arts participation on mental and psychosocial health outcomes: a randomised controlled trial of a secondary school-based mental health promotion program. *BMC Psychology*.

[19] Gao P., Li J. Y., Liu S. (2021). An introduction to key technology in artificial intelligence and big data driven e-learning and e-education. *Mobile Networks and Applications.*.

[20] Castillo L. G., Schwartz S. J. (2013). Introduction to the special issue on college student mental health. *Journal of Clinical Psychology*.

[21] Lattie E. G., Lipson S. K., Eisenberg D. (2019). Technology and college student mental health: challenges and opportunities. *Frontiers in Psychiatry*.

[22] Arnett J. J., Žukauskiene R., Sugimura K. (2014). The new life stage of emerging adulthood at ages 18-29 years: implications for mental health. *Lancet Psychiatry*.

[23] Arnett J. J. (2000). Emerging adulthood. A theory of development from the late teens through the twenties. *American Psychologist*.

[24] Kecojevic A., Basch C. H., Sullivan M., Davi N. K. (2020). The impact of the COVID-19 epidemic on mental health of undergraduate students in new jersey, cross-sectional study. *PLoS One*.

[25] Kokkinos C. M., Tsouloupas C. N., Voulgaridou I. (2022). The effects of perceived psychological, educational, and financial impact of COVID-19 pandemic on Greek university students' satisfaction with life through mental health. *Journal of Affective Disorders*.

[26] Tran L. T., Phan H. L. T., Bellgrove A. (2021). There’s a much bigger world of science than just Australia’: Australian students’ development of disciplinary knowledge, transferable skills and attributes through a new Colombo plan short-term mobility program to Japan. *International Journal of Science Education*.

[27] Miller-Graff L. E., Cater A. K., Howell K. H., Graham-Bermann S. A. (2016). Parent-child warmth as a potential mediator of childhood exposure to intimate partner violence and positive adulthood functioning. *Anxiety, Stress, and Coping*.

[28] Son C., Hegde S., Smith A., Wang X., Sasangohar F. (2020). Effects of COVID-19 on college students’ mental health in the United States: interview survey study. *Journal of Medical Internet Research*.

[29] Auerbach R. P., Alonso J., Axinn W. G. (2016). Mental disorders among college students in the World Health Organization world mental health surveys. *Psychological Medicine*.

[30] Bruffaerts R., Mortier P., Kiekens G. (2018). Mental health problems in college freshmen: prevalence and academic functioning. *Journal of Affective Disorders*.

[31] Tanaka T. (2018). Using mental imagery to manipulate the future time perspective of young adults: effects on attentional bias in relation to depressive tendencies. *Journal of Adult Development*.

[32] Luthans F., Luthans K. W., Luthans B. C. (2004). Positive psychological capital: beyond human and social capital. *Business Horizons Bloomington*.

[33] Kim S., Kweon Y. (2020). Psychological capital mediates the association between job stress and burnout of among Korean psychiatric nurses. *Health*.

[34] King R. B., Caleon I. S. (2021). School psychological capital: instrument development, validation, and prediction. *Child Indicators Research*.

[35] Rodríguez-Cifuentes F., Segura-Camacho A., García-Ael C., Topa G. (2020). The mediating role of psychological capital between motivational orientations and their organizational consequences. *International Journal of Environmental Research and Public Health*.

[36] Santisi G., Lodi E., Magnano P., Zarbo R., Zammitti A. (2020). Relationship between psychological capital and quality of life: the role of courage. *Sustainability*.

[37] Mehrabian A., Russell J. A. (1974). *An Approach to Environmental Psychology*.

[38] Bergius R. (1994). Emotion, Emotioneles Verhalten. *Dorsch Pschologisches Wörterbuch*.

[39] Rice L. L., Moffett K. W., Madupalli R. (2013). Campaign-related social networking and the political participation of college students. *Social Science Computer Review*.

[40] Olfert M. D., Barr M. L., Mathews A. E. (2022). Life of a vegetarian college student: health, lifestyle, and environmental perceptions. *Journal of American College Health*.

[41] Peacock J. (2022). Relationships between prosocial factors and college student health. *Journal of American College Health*.

[42] Bala M. O., Chehab M. A., Al-Dahshan A., Saadeh S., Al Khenji A. (2018). Violence among adolescents in Qatar: results from the global School-based student health survey, 2011. *Cureus*.

[43] Han Z., Zhang G., Zhang H. (2017). School bullying in urban China: prevalence and correlation with school climate. *International Journal of Environmental Research and Public Health*.

[44] Kowalski R. M., Limber S. P. (2013). Psychological, physical, and academic correlates of cyberbullying and traditional bullying. *The Journal of Adolescent Health : Official Publication of the Society for Adolescent Medicine*.

[45] Chen Y. (2006). *The Research on Goal Orientation of Undergraduate Future Time Perspective*.

[46] Shen A. C. (2014). Dating violence and posttraumatic stress disorder symptoms in Taiwanese college students: the roles of cultural beliefs. *Journal of Interpersonal Violence*.

[47] Fry D., Anderson J., Hidalgo R. J. T. (2016). Prevalence of violence in childhood and adolescence and the impact on educational outcomes: evidence from the 2013 Peruvian national survey on social relations. *International Health*.

[48] Tourigny M., Hebert M., Joly J., Cyr M., Baril K. (2008). Prevalence and co-occurrence of violence against children in the Quebec population. *Australian and New Zealand Journal of Public Health*.

[49] Liang L., Zheng Y., Ge Q., Zhang F. (2022). Exploration and strategy analysis of mental health education for students in sports majors in the era of artificial intelligence. *Frontiers in Psychology*.

